The article "Effect of Pulmonary Function Training with a Respirator on Functional Recovery and Quality of Life of Patients with Stroke" was published in 2022. Journal: Contrast Media Mol Imaging.

# Effect of Pulmonary Function Training with a Respirator on Functional Recovery and Quality of Life of Patients with Stroke

**DOI:** 10.1155/2022/6005914

**Published:** 2022-08-11

**Authors:** Haitang Wei, Yang Sheng, Tao Peng, Dan Yang, Qiang Zhao, Liang Xie, Zhixia Liu

**Affiliations:** Department of Rehabilitation Medicine, Wuhan Hankou Hospital, Wuhan, China

## Abstract

A stroke is a sudden onset cerebral blood circulation disorder. It occurs in patients with cerebrovascular disease due to various predisposing factors causing stenosis, occlusion, or rupture of intracerebral arteries, which, in turn, causes acute cerebral blood circulation disturbance and clinically manifests as symptoms and signs of excessive or permanent cerebral dysfunction. It can cause serious harm to patients' physical and mental health. This study aimed to evaluate the effect of Breathe-Link breathing trainers on lung function and the ability to perform activities of daily living in patients with stroke. Sixty patients with stroke were randomly divided into two groups. One group was set as the control group and received routine breathing training. The experimental group received a Breathe-Link trainer based on regular training, with rehabilitation training for 12 weeks as the time node. Respiratory muscle strength, respiratory velocity, respiratory capacity, forced vital capacity (FVC), forced expiratory volume in the first second (FEV1), and rate in the first second (FEV1/FVC) were used to evaluate the respiratory function of patients, and the Barthel index was used to evaluate the ability to perform activities of daily living. Improvements in respiratory function and daily living ability were compared between the two groups. After 12 weeks of training, respiratory muscle strength, respiratory velocity, respiratory volume, FVC, FEV1, FEV1/FVC, and Barthel index of patients in the two groups improved compared with those before training (*P* < 0.05), and the improvement in the treatment group was better than that in the control group (*P* < 0.05). Breathe-Link breathing trainers can improve lung function and the ability to perform activities of daily living in patients with stroke, and its effect is acceptable. It can be recommended for clinical use.

## 1. Introduction

Stroke refers to an acute onset, neurological deficit syndrome due to disturbance of the cerebral local blood circulation with a symptom duration of at least 24 h. The World Health Organization (WHO) developed in 1982 in Geneva the famous “Monica” protocol, a multinational monitoring protocol of cardiovascular dynamic trends and determinants, which provides precise diagnostic criteria and typing of stroke and a uniform study methodology. The results showed that the incidence of stroke ranged from 185/100000 to 700/100000. Stroke incidence rates still differed between countries, with the highest versus the lowest differing by a factor of 3 (men) and 5 (women). As a whole, the incidence of stroke is higher in Russia, Finland, Lithuania, and Beijing, China, than in Western and Northern Europe. Stroke is the main disease that endangers the health of middle-aged and elderly individuals [1]. It is characterized by high morbidity, high mortality, and high disability rates, and its incidence is increasing annually [2]. Moreover, 80% of patients have limb dysfunction, and upper limb functional recovery, especially hand function recovery, is slow [3]. It directly affects the patient's quality of daily life and brings a great mental and economic burden to the family and society. The study found that, after stroke, patients have decreased respiratory function, decreased diaphragmatic muscle contraction, decreased expiratory and inspiratory muscle strength, and airway clearance problems [4]. Breathing is closely related to posture control and body movement, and breathing function training can reduce damage to trunk stability, balance, and motor functions [5].

The article "Effect of Pulmonary Function Training with a Respirator on Functional Recovery and Quality of Life of Patients with Stroke" was published in 2022. Journal: Contrast Media Mol Imaging.

Due to functional disorders, such as limb movement, patients with stroke lie in bed for a long time, resulting in decreased respiratory muscle strength, decreased thoracic compliance, pulmonary dysfunction, and development of airway infection and pneumonia, which not only affects the recovery of neurological function but also increases the risk of another stroke [6, 7]. Current respiratory training methods mainly improve the respiratory function of patients by improving the strength of the diaphragm and other respiratory muscles [8]. However, decreased thoracic activity in patients with stroke limits the participation of the diaphragm in respiratory movement, and routine respiratory training depends on the therapist, which has high requirements for motor function, which affects the recovery of lung function to a certain extent. Breathe-Link trainers use resistance training technology, which trains not only the diaphragm but also the intercostal muscles and other auxiliary breathing muscles [9]. When inhaled, patients need to work hard to complete the resistance inspiratory action. With an increase in breathing depth, the breathing muscles undergo complete contraction and diastolic exercise. When exhaling, there is no resistance, the thoracic cavity fills and expands, and the negative pressure in the pleural cavity increases, which is conducive to lung swelling and natural discharge of air in the lung.

Respiratory training can improve patients' cough ability and prevent pulmonary infection. Pulmonary infection which is a common complication in hemiplegic patients with stroke not only hampers the rehabilitation of neurological function but also increases the risk of recurrent stroke and the case fatality rate. It was found that patients with complicated pneumonia after a stroke had five times higher case fatality rate than patients without pneumonia. Although the application and management of antibiotics and respiratory stimulants are regulated step by step, recurrent lung infections and pulmonary hypoventilation remain as difficult clinical problems. The main objective of respiratory training is to increase the strength of inspiratory and expiratory muscles in patients and improve cough capacity, promote sputum drainage, and improve respiratory function. Respiratory training may improve patient pulmonary function and activity tolerance and improve motor function. Breathing training alone can improve lung function of patients with stroke, but there are few studies on the effect of breathing trainers combined with breathing training on lung function and the living ability of patients with stroke. Given this, this study explored the effect of breathing trainers combined with breathing training on lung function and living ability of patients with stroke, which is of certain clinical innovation and provides rich treatment means for bedside treatment and a clinical basis for lung rehabilitation in patients with stroke.

The article "Effect of Pulmonary Function Training with a Respirator on Functional Recovery and Quality of Life of Patients with Stroke" was published in 2022. Journal: Contrast Media Mol Imaging.

## 2. Materials and Methods

### 2.1. Patients

Sixty patients with stroke who visited our hospital between January 2019 and January 2021 were selected. All patients met the following criteria: (1) stroke confirmed by head computed tomography or magnetic resonance imaging (imaging diagnosis: CT findings were acute hemorrhage: hyperdense; bleeding was rapid with coagulopathy: equal/high confounding density; perihematomal hypodense edema; and the hemorrhage can rupture into the ventricles); (2) first stroke, stable condition, normal consciousness level, and stable vital signs; (3) pulmonary dysfunction; and (4) autonomous breathing with inspiratory muscle training. The exclusion criteria were as follows: (1) asymptomatic lacunar cerebral infarction, transient cerebral ischemia, and reversible stroke; (2) serious cognitive or partial neglect or other functional disorders, serious anxiety, depression, or other mental disorders and inability to carry out normal intervention or evaluation; (3) severe visual impairment or hearing impairment affecting training or evaluation; and (4) heart, liver, and kidney failure, malignant tumor, gastrointestinal bleeding, and serious nervous system diseases. The study was conducted by the ethical principles outlined in the Declaration of Helsinki and Good Clinical Practice guidelines of the International Coordinating Conference. All participants and their families provided written informed consent before starting trial-related activities.

The article "Effect of Pulmonary Function Training with a Respirator on Functional Recovery and Quality of Life of Patients with Stroke" was published in 2022. Journal: Contrast Media Mol Imaging.

### 2.2. Breathing Training

Abdominal breathing: with the patient supine, the knee was placed under the pillow, so that it was relaxed. The hand was placed on the upper abdomen. The patient was instructed to breathe in slowly with the nose, exhale with the mouth, and inhale with the abdomen slowly bulging. The highest point to maintain was 2-3 s, expiratory when the navel slowly shrinks close to the lumbar spine.

Lip contraction breathing: with a comfortable position, the patient was instructed to breathe through the nose and mouth, adopt the above abdominal breathing, and pay attention to the need to do whistling when exhaling. Diaphragm resistance training: according to the patient's situation to take the appropriate position, abdominal breathing, inhalation in the patient's upper abdomen to apply resistance, and exhalation to remove resistance were performed.

Inspiratory muscle training: cough training: the specific operation includes two normal breaths and the last forcible cough.

Lateral thoracic breathing: with a comfortable position, both the hands were placed on the lower chest. The patient's breathing rhythm was observed, and the patient was instructed to resist external force to expand the thoracic cavity when inhaling and at the end of expiration to exert power to exhale more fully. The abovementioned training was 5–10 min each time, twice a day, 10 times a week, for 12 weeks.

### 2.3. Breathe-Link Training Instrument

The training time was arranged for 1-2 h after meals. During training, patients should sit or stand in an upright position to allow them to relax. Patients with hand strength were required to hold the Breathe-Link trainer by themselves. Patients without hand strength should be assisted by nurses in holding the Breathe-Link trainer; then, the Breathe-Link trainer was connected to a computer and turned on in the inspiratory muscle training app. It is placed inside the mouth with the lips wrapped airtight, and the middle is grabbed between upper and lower teeth, according to the prompt to guide patients with inspiratory training, as much as possible before the suction in gas is exhaled. Effectively quick inspiration was performed, with breathing from slow to fast, allowing thoracic expansion. Then, as the lung gas passed through the mouthpieces, the chest and shoulder muscles were relaxed. The training was performed 30 times, twice a day, and arranged after breakfast and lunch for 4 weeks.

The article "Effect of Pulmonary Function Training with a Respirator on Functional Recovery and Quality of Life of Patients with Stroke" was published in 2022. Journal: Contrast Media Mol Imaging.

### 2.4. Respiratory Function Assessment

Respiratory muscle strength reflects the strength of the patient's respiratory muscle during breathing; flow rate (flow), the volume of breathing gas per unit time, reflects respiratory capacity and airway patency; and volume, the volume of breathing gas, mainly reflects the ability to breathe. The following parameters were evaluated using a pulmonary function tester: forced vital capacity (FVC), forced expiratory volume in the first second (FEV1), and FEV1/FVC.

### 2.5. Activities of Daily Living (ADLs)

ADLs were assessed using the Barthel index. The scoring criteria were as follows: 1 point = you can do it yourself; 2 points = some difficulties, can do it on their own; 3 points = need help; 4 = impossible at all; 1 is when the patient never does it but is competent, 2 is when the patient never does it but has difficulty doing it but does not need help, 3 is when the patient never does it but needs help doing it, and 4 is when the patient never does it and cannot do it. A normal score ranged from 20 to 80, and a score < 20 indicated cognitive impairment.

### 2.6. Statistical Analysis

Data analyses were performed using SPSS 22.0 (IBM Corp., Armonk, NY, USA). Data are presented as measured values ± standard deviation and number data (*n* (%)) and were adopted for the experimental data analysis. Group comparisons using paired *t*-tests were performed using GraphPad Prism 8.0 (GraphPad Software, Inc., La Jolla, CA, USA). Multiple group comparisons were performed using analysis of variance. The significance level was set at a *P* value < 0.05.

## 3. Results

### 3.1. Patients

Sixty patients were randomly divided into the experimental and control groups, with 30 patients in each group. In the experimental group, there were 15 men and 15 women with an age of (48.1 ± 4.1) years, and the disease duration was 3.9 ± 1.4 months. Among these patients, 17 had a cerebral hemorrhage and 13 had cerebral infarction. The control group comprised 15 men and 15 women. The age was 47.8 ± 4.4 years, and the disease duration was 3.8 ± 1.1 months. Among them, cerebral hemorrhage occurred in 18 patients and cerebral infarction in 12 patients. There were no significant differences in sex or disease between the two groups (*P* > 0.05).

### 3.2. Respiratory Function before and after Treatment

The results showed that after treatment, the respiratory muscle strength, flow rate, and volume of the two groups were higher than those before treatment (*P* < 0.05). In addition, the increase was more significant in the experimental group than in the control group (*P* < 0.05), as shown in Table 1.

The article "Effect of Pulmonary Function Training with a Respirator on Functional Recovery and Quality of Life of Patients with Stroke" was published in 2022. Journal: Contrast Media Mol Imaging.

### 3.3. Lung Function before and after Treatment

After treatment, FVC, FEV1, and FEV1/FVC in both groups improved compared with those before treatment (*P* < 0.05). In addition, the experimental group showed greater improvement than the control group (*P* < 0.05). The results showed that the respiratory trainer effectively enhanced the lung function of patients after treatment, as shown in Table 2.

### 3.4. ADL before and after Treatment

After treatment, the ADL scores in both groups improved compared with those before treatment (*P* < 0.05). In addition, the improvement was more pronounced in the treatment group than in the control group (*P* < 0.05), indicating an acceptable effect of the breathing training equipment, as shown in Table 3.

## 4. Discussion

Due to impairment of the brain nerve and weakening of nerve control, the trunk and core mobilization ability of the body is weakened in patients with stroke, resulting in trunk muscle dysfunction of different degrees, balance dysfunction, and other abnormalities, which are affected by the compensatory movement of the healthy side, causing body tilt and adverse left and right asymmetric limb movements [10–12]. The stability of the human trunk core is accomplished by the precise control and normal contraction of core-related muscle groups, such as the trunk and pelvis, mainly including the abdominal, lumbar, and back muscles [13, 14]. When the body is affected by external forces or changes in itself and needs to readjust balance, the normal path is through the rectus abdominis, external oblique, and trapezius muscles, and the latissimus dorsi and erector spinae muscles can achieve rapid reactive contraction, which can maintain posture and stabilize the trunk in human movement [15, 16]. In the training of patients with stroke, core muscle group training of the trunk is beneficial to improve coordination and control ability among various motor muscle groups of the body, while the contraction and stability of the trunk core are limb movement, creating a fulcrum and coordinating body movement so that the power of transmission and control to reach the optimal level improve the efficiency of movement, and upper limb movement recovery has a positive role and can improve the patient's daily activities [17–19].

Studies at home and abroad have found that respiratory dysfunction can affect the trunk control and balance function of patients with stroke and has a certain effect on the recovery of limb function in patients [20]. In patients with stroke, respiratory training can improve respiratory function, respiratory muscle strength, and cough expectoration [21]. Improved trunk control and balance function in the sitting position of patients with stroke by improving trunk strength [9]. Respiratory muscles play important roles in core and trunk stability. Core stability training based on strengthening the movement control of respiratory muscles significantly improves the movement control ability of the body [5]. In this study, patients in the control group underwent respiratory training. After 12 weeks of treatment, the patients' respiratory and lung functions were better than before, indicating that this method has a good clinical effect.

The article "Effect of Pulmonary Function Training with a Respirator on Functional Recovery and Quality of Life of Patients with Stroke" was published in 2022. Journal: Contrast Media Mol Imaging.

Breathe-Link trainers have low requirements for patients' body functions, and patients can see changes in related parameters during training, thus improving their enthusiasm and compliance with training [9]. In this study, we found that after treatment, respiratory muscle strength, flow rate, and volume of breath were enhanced, and lung function was significantly improved in the experimental group compared with that before treatment. In addition, in this study, the combination of Breathe-Link trainer and breathing training effectively improved the treatment efficiency in patients. After treatment, compared with a single breathing training, the lung function of the experimental group is significantly improved than that of the control group. The improvement of lung function lays a foundation for the rehabilitation of limb movement and other functions of patients, which can promote their ability to perform ADLs. This study showed that, after 12 weeks of treatment, ADL in both groups increased, and ADL in the experimental group was significantly higher than that in the control group (*P* < 0.05). These results suggest that Breathe-Link trainers combined with breathing training could improve lung function and the ability to perform ADLs in patients [22].

Due to the limitation of observation time, the sample size in this study was insufficient, and the long-term efficacy of respiratory training was not followed, which had a certain impact on the accuracy of observation results. This will be explored in future studies, in which we will expand the sample size and extend the follow-up duration.

## 5. Conclusion

A Breathe-Link trainer combined with breathing training can improve lung function and the ability to perform ADLs. In addition, improvements in lung function may increase ADLs in patients.

## Figures and Tables

**Table 1:** Comparison of respiratory function between the two groups before and after treatment.

Group	Respiratory muscle strength (mmHg)		Flow rate (L/s)		Capacity (L)	
	Before 12 weeks	After 12 weeks	Before 12 weeks	After 12 weeks	Before 12 weeks	After 12 weeks
Experimental group	30.6 ± 0.4	41.1 ± 0.5^∗^^**#**^	1.5 ± 0.1	1.9 ± 0.1^∗^^**#**^	1.2 ± 0.4	1.5 ± 0.1^∗^^**#**^
Control group	30.7 ± 0.4	46.5 ± 1.1^∗^	1.5 ± 0.3	2.8 ± 0.1^∗^	1.1 ± 0.3	1.8 ± 0.1^∗^

1 mmHg = 0.133 kPa. ^**#**^Compared with the control group, *P* < 0.05; ^∗^compared with 12 weeks before, *P* < 0.05.

The article "Effect of Pulmonary Function Training with a Respirator on Functional Recovery and Quality of Life of Patients with Stroke" was published in 2022. Journal: Contrast Media Mol Imaging.

**Table 2:** Comparison of pulmonary function tester parameters before and after treatment.

Group	FVC (L)		FEV1 (L)		FEV1/FVC (%)	
	Before 12 weeks	After 12 weeks	Before 12 weeks	After 12 weeks	Before 12 weeks	After 12 weeks
Experimental group	1.9 ± 0.1	3.3 ± 0.1^∗^^**#**^	1.5 ± 0.2	2.6 ± 0.2^∗^^**#**^	62.3 ± 8.3	74.9 ± 8.7^∗^^**#**^
Control group	1.9 ± 0.1	2.2 ± 0.1^∗^	1.4 ± 0.1	1.5 ± 0.1^∗^	62.4 ± 8.7	70.1 ± 8.2^∗^

^**#**^Compared with the control group, *P* < 0.05. ^∗^Compared with 12 weeks before, *P* < 0.05. FVC, forced vital capacity; FEV, forced expiratory volume in the first second.

**Table 3:** ADL before and after treatment.

Group	Before 12 weeks	After 12 weeks
Experimental group	42.1 ± 0.6	63.8 ± 3.2^∗^
Control group	42.1 ± 2.2	57.5 ± 5.7^∗^^**#**^

^**#**^Compared with the control group, *P* < 0.05. ^∗^Compared with 12 weeks before, *P* < 0.05.

## Data Availability

The data used to support the findings of this study are available from the corresponding author upon request.
